# Corrective Mechanism Aftermath Surgical Treatment of Spine Deformity due to Scoliosis: A Systematic Review of Finite Element Studies

**DOI:** 10.1155/2022/5147221

**Published:** 2022-07-18

**Authors:** Kavita Gunasekaran, Khairul Salleh Basaruddin, Nor Amalina Muhayudin, Abdul Razak Sulaiman

**Affiliations:** ^1^Faculty of Mechanical Engineering Technology, Universiti Malaysia Perlis, 02600 Pauh Putra, Perlis, Malaysia; ^2^Medical Devices and Health Sciences, Sports Engineering Research Center (SERC), Universiti Malaysia Perlis, 02600 Pauh Putra, Perlis, Malaysia; ^3^Department of Orthopaedics, School of Medical Science, Universiti Sains Malaysia, 16150 Kubang Kerian, Kelantan, Malaysia

## Abstract

This paper presents a systematic study in reviewing the application of finite element method for the analysis of correction mechanism of spine deformity due to scoliosis. The study is aimed at systematically (1) reviewing the use of finite element analysis in spine deformity case, (2) reviewing the modelling of pedicle screw and rod system in scoliosis surgery, and (3) analysing and discussing gap between the studies. Using the restricted key phrases, the review gathered studies from 2001 to 2021 from various electronic databases (Scopus, ScienceDirect, PubMed, Medline, and WorldCAT). Studies were included if they reported a finite element study on spine deformity. Studies that did not fully disclose their methodology and results had significant discrepancies, not published in English or not yet published were all disqualified. Regardless of inconsistencies in the methodological design of the studies, the quality of all papers was above the acceptable level. A total of fifteen manuscripts were considered for inclusion and were given a comprehensive review. This study indicates that analysing the forces acting on the spine, as well as the interrelationship between the force, stress, and degree of correction (which measured as the Cobb angle), could help to improve the corrective mechanism procedure of spine deformity. Pedicle screws and its placement strategies are also important as it influence the corrective forces for scoliosis treatment. Hence, the findings of this study could potentially be used as a guidance to develop a reliable finite element analysis that can predict the biomechanics responses during the corrective spine deformity treatment.

## 1. Introduction

Scoliosis is a three-dimensional (3D) spinal deformity characterised by axial vertebral rotation. The Cobb angle value is used to determine the severity of a scoliotic deformity. The Cobb angle is the maximum angle made in the frontal plane by two lines drawn parallel to the endplates of scoliotic vertebrae. Surgical treatment with implant fixation is used when the Cobb angle is more than 50° [1]. There are several surgical procedures that have evolved to be more advanced in applying the three-dimensional corrective forces for the correction of severe scoliotic deformity. Cotrel and Dubousset's (CD) rod derotation technique, ventral derotation spondylodesis (VDS), Halm–Zielke instrumentation (HZI), simultaneous dual rod rotation method (SDRRT), direct incremental segmental translation (DIST), and others are examples of these procedures [1, 2]. These surgical therapies for severe scoliosis need the use of surgical methods to secure implanted devices such as rods, screws, hooks, and wires. For example, the anterior single rod correction procedure in Figure 1 involves removing the malformed intervertebral discs, implanting material to stimulate intervertebral joint fusion, and attaching metal rods to the spinal vertebrae [3] as spine deformity correction procedure.

The usage of computer simulations of the spine has skyrocketed in the last two decades. Computational techniques, notably finite element method (FEM), have previously been demonstrated to be effective in analysing the mechanics of the scoliotic spine during surgery [3]. For instance, Aubin et al. [4] created a model of the spine that had rigid bodies that represented the thoracic and lumbar vertebrae seen on intraoperative radiographs, as well as flexible parts that represented the intervertebral structures. Developing an optimal system of corrective force for an individual scoliosis patient via trial and error during surgery is actually unrealistic. Hence, FEM has been used to simulate surgical process changes and predicts the three-dimensional outcome in terms of deformity treatment and build flexibility. The FEM used in scoliosis research was divided into four groups based on model complexity: reflective simple variants of beam element-based models, representative complicated versions of beam element-based models, representative segmental volumetric models, and representative extensive volumetric models, according to the previous study [5].

By developing FEM, the relationships between the magnitude of corrective forces, number of screws, screw placement configuration, and degree of correction can be further elucidated [2]. Actually, the well-developed FEM of the spine allows for more complete assessments of internal stress distribution [6]. The studies of internal stress distributions and hypothetical scenarios cannot be properly examined without the help of real patient records, which is a possible drawback of rigid body modelling and patient-based FEM design.

Scoliosis correction aims to distort and restore the scoliotic spine to its original shape without inflicting injury or neurological complications. This could be accomplished by using implant rods and screws to impart appropriate correction forces to the spine. To obtain the optimum correction, the corrective forces required to rectify the deformity must be adequate [6]. Despite the fact that the number of patients was small, there was a growing correlation between the applied force and the degree of correction. Nevertheless, because of the rotating device is only linked to the implant rod, the correction forces acting at every screw were quite hard to be measured.

## 2. Methods

### 2.1. Search Strategy

Database search through the internet performed in November 2021 was restricted to the last twenty years of publication in Scopus (2001-2021), ScienceDirect (2001-2021), WorldCAT (2001-2021), PubMed (2001-2021), and Medline (2001-2021). The key MESH terms included “correction,” “spine,” and “deformity.” A thorough search was also conducted using the additional keyword search query: “finite element.” This extra manual search was implemented by manual screening conducted for relevant articles based on the reference lists of the retrieved articles. To rule out the likelihood of those items being overlooked, an additional search was conducted. All of the articles were retrieved and checked to ensure that the database search results were accurate and related to other articles. The ultimate decision was drawn in order to keep our findings within the scope of the papers.

### 2.2. Inclusion/Exclusion Criteria

From the electronic databases, only full-text articles in English were chosen. If there was a disagreement about an article during the screening process, it was debated to reach a consensus. Articles on studies focusing on corrective deformed scoliosis were included in the titles and abstracts screening procedure. The following criteria were used to evaluate articles: (1) rod and pedicle screw system, (2) Cobb angle, and (3) finite element analysis, full nonclinical articles. There were no restrictions on the participants' age, gender, BMI, or medical history. Articles by the same author were double-checked to ensure there were no duplicates.

### 2.3. Review Process

Two reviewers (K.G. and K.S.B.) screened the search results according to the inclusion criteria. After the screening procedure, the final articles were extracted and separated from duplicated articles in several databases. Duplicate articles were eliminated from various databases. The eligibility criteria were initially applied to the titles and abstracts of the papers that were chosen. A full-text review was undertaken if the title and abstract did not give enough information in the article screening procedure. To avoid misinterpretation, rejected items were rescreened.

### 2.4. Assessment of Methodological Quality

The papers were reviewed and analysed using a systematic quality approach that helped to evaluate the quality of the articles identified, as well as extracting the most relevant information from those publications. There are no standardised methods for evaluating the reliability and credibility of each of the articles examined aside than the processes provided in this study. To evaluate credibility, 13 questions were adapted from Azizan et al. [7] and Ku et al. [8]. Few questions were had to drop as they are not justifying to spine deformity and its correction mechanism. At the same time, some of the questions were later altered according to FEA. Each question was given a score of “2” if the answer satisfied the standard questions, and a score of “1” if the information was limited. If no information was provided, the questions were marked with “0” or “no,” while questions that were not applicable were marked with “NA.” The 13 questions are as follows:

1. Is the study's objective stated in a clear and concise manner?
2. Is the study design outlined in detail?
3. Are the patients'/models' characteristics and details clearly provided?
4. Is the process of geometrical model development clearly explained?
5. Is the convergence test in the study clearly stated?
6. Is the boundary condition clearly described?
7. Are the appropriate mathematical models used to calculate parameters?
8. Are the mechanical properties of the model distinctly defined?
9. Are appropriate numerical methods used in data analysis clearly defined?
10. Is the predicted numerical value appropriately verified or validated?
11. Is the key outcome measure mentioned clearly?
12. Are the study's limitations disclosed clearly?
13. Is the study's conclusion conveyed in a clear and concise manner?

## 3. Results

### 3.1. Primary Search Results

Since the number of findings was limited in terms of quantity of information and the amount of materials available, the authors then conducted full-text reviews of articles. After a thorough screening process, twenty-two retrieved articles were finalised.  Figure 2 shows the systematic review process of the present study. A total of 967 items were found after the database screening procedure. 81 of these items, however, were found duplicates and were removed. The relevancy of the studies undertaken was determined by looking at the titles and abstracts, and then, 602 publications were eliminated. Additional screening was carried out by reading the rest of the article's content in order to ascertain the study's goal based on the standard parameters that was assessed. After removing another 42 articles, there were 15 articles that meet all the criteria and were further reviewed.

### 3.2. Analysed Data Quality

Table 1 shows the quality ratings of the 15 articles that were assessed. The reviewed papers have a quality score ranging from 80% to 96%. Articles with a score of more than 85% are regarded good because they provide answer for all thirteen questions. These publications offered detailed information about their objectives, study design, key findings, and conclusion [1, 3, 9]. The remaining eleven studies fulfilled at minimum 70% to 90% of the questions [6, 10]–[11]. Other elements that could have aided in the comprehension of the questions were not considered in this review.

### 3.3. Participant Characteristics

Table 2 shows a list of physical characteristics and anthropometric factors from 15 articles. The majority of the participants were young people, with only a few adults of average age. Nine studies involved adolescences (aged between 10 and 19) [1, 3, 9, 11, 12, 14, 15, 17], two articles assessed middle-aged individuals (age range from 30–59) [10, 19], and none of the articles involved elderly persons (aged 60 and above). The number of participants in the evaluated publications varied, with the highest number being 20 peoples and seven articles keeping one as patient data for their investigation [6, 9, 11, 12, 16, 18, 19]. Four articles provide no anthropometric data of tested participants as those studies used spine finite element models [6, 16, 18, 20]. The participants were also categorised into presurgical [1, 2] and postsurgical patients [3, 12].

### 3.4. Finite Element Modelling

By conducting an exhaustive search for all published papers, a systematic review aims to minimise the incidence of bias. The modelling parameters in FEA, such as loads and boundary conditions, element types and sizes, geometrical model, type of material, and mechanical properties, have a significant influence on prognostic accuracy. These variables have an impact on the simulation's predictive accuracy and should be considered when evaluating the results and conclusions.  Table 3 shows finite element modelling variables that were used by the reviewed articles on the corrective mechanism of spine deformity due to scoliosis. These data can provide additional information on the simulations, allowing for replication and comparison.

Ten out of fifteen studies used ANSYS software for FEA studies [1, 2, 6, 9, 15, 18, 19]. Whereas Abolaeha et al., Little et al., and Guan et al. used ABAQUS software [3, 12, 18]. Wang et al. mentioned only radiographic software used for his FEA studies [20]. Special mention to Chen et al. [19] where Solidworks was the primary software for FEA studies where the pedicle screws created based on the imported blueprint then into Hypermesh and assembled into scoliotic spine FE model. Elements are the basic building block of FEA. Several authors used 10 node tetrahedral solid elements [1, 2, 9, 11, 14]. However, Wang et al. [15] and Guan et al. [18] used hexahedron elements. Moreover, beam elements for vertebral and pelvic sections, tension-only cable elements for ligaments, surface contact elements for articular facets, and modified beam elements are all included in FE model by Dumas et al. [10].

In order to produce an accurate reconstruction, the image quality is critical. To develop a rebuilt model as accurate as possible, it can be seen that the models in most of the studies were created from computed tomography (CT) scan images that was widely used by the researchers [1, 3, 6, 9–12, 15, 16, 18], either directly or via a previous model's scaling. Meanwhile, only Wang et al. [13] used ADAMS 2005 software (Mechanical Dynamics Inc., Ann Arbor, MI) and the ADAMS Software Development Kit (SDK). Finite analysis has been shown to be useful in understanding the aetiology of scoliosis in these models. To ensure that the model performs realistically, the produced FEM must be tested against existing scientific results on motion and material properties.

As for the material, titanium alloy was widely used for both rod and screws compared to cobalt chromium which also has elastoplastic properties [1, 3, 12, 15, 18, 19]. Abolaeha et al. [12] used stainless steel that also has elastoplastic material behaviour as aluminium alloy. Some authors used both aluminium alloy and cobalt for screws and rod, respectively [3, 17]. As for the mechanical properties, the range of elastic modulus for rod is between 105 GPa to 213 GPa [1, 3, 6, 15, 17, 20].

Modern segmental spinal instrumentation systems are used to execute a variety of deformity correction techniques, including vertebral translation, rod derotation, direct vertebral derotation, and in situ rod contouring, all of which have been thoroughly studied. Dumas et al. [10] introduced situ contouring technique in his studies. Whereas Abolaeha et al. [12] used spinal growth rod instrumentation, an early onset scoliosis management method, and emerging technology that treating scoliosis without fusion hold the exciting prospect of a new paradigm in spinal deformity care. Salmingo et al. in their both studies and Abe et al. [1, 2, 14] used simultaneous double rod rotation technique (SDRRT) surgical technique with rods and polyaxial pedicle screws. Wang et al. [13] studied a posterior instrumentation using monoaxial pedicle screws, whereas Chen et al. [19] presented a procedure that includes rod derotation on the concave side and rod implantation on the convex side for strengthening.

Setting boundary condition is an important procedure that has to be done while set up simulation process of the finite element analysis. Dumas et al. [10] set displacement to the model as one of the boundary conditions. Displacement by means, the 3D motion of T1 with regards to the pelvis was computed between the bending test measurements and the standing position measurements. Force that could be directly applied was also set as the boundary conditions of the surgical manoeuvre.

There are several studies that have set the boundary conditions as constraining motions of particular vertebra. Balamurugan et al. [16] set the L5 vertebra as constrained from all degrees of freedom, and a compressive force of 50 N along the *Z*-axis was applied on T1 vertebra for the analysis. On the other hand, in the Salmingo et al. works [1, 2], the boundary condition was set considering the manner of rod fixation during the surgical treatment. The screws' coordinates were reoriented such that the most superior screw coincides with the *z*-axis (located on top of the most inferior screw) because each patient has different implant rod orientation and fixation levels. The most inferior screw at the end of the rod was fixed in all translations but free to rotate. The most superior screw was also fixed except that it was free to move along the superior direction only. The same practice was applied by Guan et al. [17] in their research where the boundary conditions were included as a fixed pelvis in rotation translation, and *T*1 was limited to transverse plan movements. Zhang et al. [9] also set constraint on the displacement and rotation of all nodes on the base of the L5 vertebral body in all directions. However, there is no thoracic regions vertebra was included to set as boundary conditions.

Apart from abovementioned boundary conditions, the contact between rod and screw surface was also introduced by Little et al. [3] in their research. A “no separation” normal contact and frictionless tangential contact definition were defined between the screw head and the surface along the rod during surgery.

Researchers, on the other hand, have developed a variety of approaches to model the loading circumstances and limitations that are relevant to the corrective spine deformity process. Commonly, to achieve the desired correction, the force required to rectify the deformity must be significant. After a set of iterations with the force optimization method, the corrective forces acting on the implant rod were obtained [1]. Salmingo et al. [1, 2] analysed forces of screws set with initial values of zero before surgery on each screw's matching point on the rod geometry. According to Wang et al. [15], Balamurugan et al. [17], Abolaeha et al. [12], and He et al. [11] studies, load was applied to the upper region of the vertebrae for observation of stress distribution. This was applied as boundary condition.

### 3.5. Variability in Measured Parameters

The output and findings of the parameters are summarised in Table 4. The focus of this data analysis is to look at the relevant biomechanical criteria that are often used to identify FEA and/or have clinical value.

Most of the articles focused on the influence of Cobb angles which is to indicate magnitude of spine deformity except for two articles which are Balamurugan et al. [17] and He et al. [11] that concentrated on the effect of surgery on deformity treatment in a scoliotic spine. Preoperative and postoperative main curves were described in four different investigations after follow-up period, and the degree of correction varies from 14° to 70° [1, 3, 12].

In this review, scoliosis in several planes' views such as lateral, sagittal, axial, frontal, transverse, and coronal can be observed. Most of the authors studied scoliosis deformity in both sagittal [2, 9, 12, 13, 18] and coronal plane [3, 9, 11, 15, 16, 18]. However, Salmingo et al. and Zhang et al. focused on frontal plane [1, 9].  Figure 3 shows an example of a lateral displacement of the spine from the midline in the coronal (frontal) plane, decreased curvature in the thoracic region in the sagittal (side) plane and rotation in the axial plane.

Most of the authors carried out force analysis during the treatment of the spinal deformity and growth periods, on the rods and the spine for their studies [1, 3, 6, 12, 14, 16, 19]. Few of them created stress profile to understand the stress concentration profile on the vertebra and disc under different loads [1, 9, 11, 17]. Meanwhile, Dumas et al. [10] focused on rod rotation analysis on lateral, sagittal, and axial plane, and Wang et al. [15] demonstrated ranges of motion for L2 to L5 under various loading scenarios.

## 4. Discussion

### 4.1. Quality of Search

The aim of this systematic review was to analyse the biomechanical characteristics and parameters that are typically used in finite element analysis to investigate the corrective mechanism of scoliosis-related spine deformity. Understanding the corrective mechanism requires a comprehensive analysis on the parameters used in each investigation. In the present study, fifteen articles were included for the extensive review. In the reviewed studies, participants' characteristics, Cobb angle, pedicle screw systems, and biomechanical responses can be further discussed.

### 4.2. Effect of Deformity Angles on Spine Corrective Forces and Stresses

The simulated corrected Cobb angle is usually attributed to the clinically established postoperative Cobb angle in the immediate postoperative period. This could provide the models' accuracy in forecasting the change in coronal deformity following surgery. The Cobb angle which is used for comparison of deformity level is the maximum angle that can be projected between the upper and lower endplates of the scoliotic curve. To treat and prevent worsening deformity in severe cases of scoliosis (Cobb angle more than 45°-50°), surgical instrumentation or, in some cases, spinal fusion is sometimes utilised. Developing an optimum method of corrective force and predicting surgically imposed contact stresses between adjacent vertebral endplates for scoliosis patient during surgery through practical experiment is quite difficult. Hence, FEA can be used to model different surgical procedures and anticipate the three-dimensional results in the form of deformity correction and construct flexibility.  Table 3 covers the variables involved in FEA studies.

Understanding and analysing the forces acting on the spine, as well as the interrelationship between both the force and the Cobb angle, will enable us to advance with improved systems [12]. According to Abolaeha et al., the resultant Cobb angles are inversely proportional to the progression of growth, rod lengths, and distraction force during a two-year period. To assess the forces required to treat scoliosis, Salmingo et al. [1] created an elastoplastic FEM. Based on differences in implanted geometry before and after surgery, the three-dimensional forces required to deform a rod were calculated. The instrumented spine's at the lowest level experienced the highest forces.

Using the same FE model, Salmingo et al. continued to study the relationship between the magnitude of corrective forces and the degree of correction, which they measured changes of Cobb angle [2]. Actually, these values can be obtained by calculating the difference between preoperative and postoperative Cobb angle. They claimed that the degree of correction and the corrective forces operating on the rod were unrelated too. They also suggested that other factors, such as screw implantation arrangement and spine rigidity, may be linked to scoliosis repair.

However, from the study carried out by Little et al. [3] revealed that increasing the simulated intraoperative forces caused the anticipated corrected Cobb angle to decrease. Force, geometry (human anatomical), and tissue stress are involved in coronal plane deformity treatment. These are the most significant considerations in getting the best possible correction for a patient with the least amount of risk of high stresses on the spinal tissues, which could lead to implant-related problems.

After adding a growing rod, Abolaeha et al. [12] created a scoliotic spine FEM to model the spine growth over a two-year period. Based on the analysis, the pressures required to induce the correct Cobb angle changes are identical to those seen in patients. To distribute the load, the rod was linked to both vertebrae in the pair, which is identical to the present surgical insertion process. At the time of the original operation, it was expected that the deformity angle would be rectified by 50%. Following the initial operation, invasive lengthening treatments (similarly referred as distractions) were conducted every six months over a year to keep up with the growth of the spine.

Meanwhile, Guan et al. [18] concluded that whenever 3D correction forces rose, the thoracolumbar segment's Cobb angle steadily reduced, and the vertebral body's rotation angle lowered as well. The combined force correction effects were even higher. When correction forces were applied, stress at intervertebral discs in the distorted region changed drastically. Essentially, during scoliosis surgery, corrective force cannot be applied to the spinal implant beyond the anchor holding strength limit. If the corrective force exceeds the anchor's strength, the implant may break or the bone may fracture, resulting in “screw ploughing.” Destabilization of the spinal segment by releasing soft tissue or the facet joint could be more critical than using an excessive correction manoeuvre with rigid implant to avoid implant fracture or pedicle rupture during a more severe curve correction procedure [14].

### 4.3. Analysis of Pedicle Screws and Implant Rod System due to Spine Deformity

For the treatment of spinal malformations, pedicle screw fixation has become a common surgical instrumentation approach. The better bone-implant connection allows surgeons to diagnose more corrective movements and employ larger correction pressures when translating and derotating the deformed spine. Hence, pedicle screws and its placement strategies are important as it has a minor influence on the curve correction scoliosis treatment [14]. In recent years, fewer screws have been used in scoliosis surgery for cost considerations, and correction rates have been reported as being similar between the less density group and the high-density group. For instance, Salmingo et al. [2] carried out a study by increase in absolute number of implant screws which resulted in reduction of the magnitude of corrective forces and did not give a greater degree of correction, and it was hypothesised that additional screws might prolong the surgery and result in more blood loss for the patients.

On the contrary, Clin et al. [16] discovered that reducing the number of screws raised the postoperative stresses that each screw could withstand, but that the influence on potential problems has to be investigated further. In their investigation, they found that independent of screw type, both high-density and low-density implant designs achieved comparable coronal correction and shared corrective forces equally well. Increased degrees of freedom of the screw head were also discovered to decrease the potential to cure coronal deformity while generating reduced bone-screw forces.

Theoretically, a greater number of implantations might give higher correction forces, resulting in better coronal and sagittal plane correction rates. A screw–rod connection which provides degrees of freedom, on the other hand, may make it difficult to perform the desired manoeuvres [21]. In addition, other variables such as curve flexibility, surgeon-specific objectives, and procedures may also play a role in the contradictory findings [19]. Wang et al. [20] used three forms of screws namely monoaxial, polyaxial, and dorsoaxial pedicle screws for their study. At each step, external forces must be raised until the rods can easily lock into the screw head saddles, which is linked to minimum “true corrective forces” (TCF) and little to no “Extra Forces” (EF) available to deliver the desired correction. The results showed that the dorsoaxial screws allowed for the least amount of EF to be created while forcing in order to make it certain appropriate rod seating and locking at all pedicle screws for corrective deformity correction. Clin et al. [16] claimed that lowering implant density by 30% permitted almost same degree of coronal correction as a fully instrumented construct irrespective of pedicle screw type, but that the influence on potential complications has to be investigated further.

He et al. [11] also claimed as pedicle-screw-rod system (PSRS) has always been regarded as the gold standard for the scoliosis treatment even though it has its own limitations. PSRS has several advantages, including rigorous fixation of deformities, increased osseous fusion, and a lower rate of pseudarthrosis. Front and mid columns are protected by rigid fixing, which counteracts eccentric stress. In addition, the fusion rate of stiff fixing is higher than that of semirigid fixing or no fixing. High stiffness, on the other hand, promotes fast scoliosis stability and minimises the physiological stress on the deformed vertebra.

Despite the fact that in recent years, the quality of studies in this field has improved, this review underlines the present literatures lack of regular use of standardised measures of end results and methodologies for preoperative and postoperative assessment. This standard should be broadened to include procedures for classifying and reporting complications. For example, past research has shown that excessive correction forces might could result in implant or bone fractures, which could result in screw extraction from the vertebra. As a result, gaining a better knowledge of scoliosis correction biomechanics necessitates an examination of corrective forces acting on the deformed rod [1].

Once the implant has been installed, the stress is centred on the two ends of the vertebral body, the rod, and the pedicle screw, resulting in a stress shielding effect. The stress shielding reduces the pressure on the intermediate vertebral body, and it just may result in bone loss and osteoporosis. Another limitation is that the cephalic and posterior sides of fixed segments have their rotation centres shifted. Because of these disadvantages, some orthopaedics professionals and researchers recommend using biodegradable or internal fixing materials with a low Young's modulus [11].

Another notable highlight is lack of studies by previous researchers which focus only one specific region either it is lumbar or thoracolumbar region. Most of the researchers either involves whole spine region or mostly thoracolumbar region for their studies ([1, 2, 9, 11, 12, 15, 17, 20]. Actually, between thoracic and lumbar vertebrae, there are changes in transverse process bone mass and anatomical structure [11]. As a result, more research involving patients' thoracic regions is required. The search method was confined to English-language articles, which is a limitation of the study. To discover articles, only five databases were used, and it is possible that some articles were overlooked. For the missing relevant articles, a manual search was conducted.

## 5. Conclusions

The present review highlights fifteen articles related to corrective mechanism of spine deformity that is published from 2001 until 2021. The correction mechanism, pedicle screw, rod system, Cobb angle, and other variable characteristics related to scoliosis surgery on patients' bodies were the subject of this review. The collected data were able to furnish basic details about the simulations as well as some variables that may affect the predictive accuracy of the simulation. However, insufficient information in certain aspects prevents the analysis of related measured variables. There are various aspects that associated to scoliotic patients such as muscular activation, spine rigidity, deformity severity, the amount of stress that an internal fixation could withstand, and inter-individual differences have yet to be investigated. Insufficient information prevents the analysis of related measured variables. Hence, to improve and provide a better knowledge of the finite element approach for the analysis of correction mechanisms of spine deformity due to scoliosis, further research is needed in the areas stated above.

## Figures and Tables

**Figure 1:** Sample of spine radiographs, (a) preoperatively and (b) postoperatively with having a single rod (anterior procedure) [3].

**Figure 2:** The research selection procedure from the reviewed articles.

**Figure 3:** A spine with scoliosis with coronal, sagittal, and axial plane views [5].

**Table 1:** Overall score based on the articles that were reviewed.

Authors and years	Questions													Overall score	Overall %
	1	2	3	4	5	6	7	8	9	10	11	12	13		
Dumas et al. [10]	2	2	1	1	1	2	0	0	1	2	2	0	2	16/20	80.0
Abolaeha et al. [12]	2	2	NA	1	1	0	1	2	2	2	2	0	2	18/20	90.0
Salmingo et al. [1]	2	2	2	2	1	1	2	2	2	2	2	2	1	23/26	88.5
Wang et al. [13]	2	2	0	0	1	0	0	2	2	2	2	2	2	17/18	94.4
Driscoll et al. [6]	2	1	0	0	NA	0	1	2	2	2	2	0	2	14/16	87.5
Salmingo et al. [2]	*2*	2	1	1	1	2	2	2	2	2	2	2	2	23/26	88.5
Little et al. [3]	*2*	2	1	1	2	2	2	1	2	2	2	2	2	23/26	88.5
Abe et al. [14]	2	2	2	2	NA	0	2	1	2	2	2	1	2	20/22	91.0
Wang et al. [15]	2	2	2	2	1	0	1	2	2	2	2	2	1	21/24	87.5
Clin et al. [16]	2	2	2	2	NA	0	2	1	2	2	2	2	2	21/22	95.5
Balamurugan et al. [17]	2	2	0	0	NA	0	2	2	2	1	2	0	2	14/16	87.5
Guan et al. [18]	2	2	2	2	2	2	2	2	2	2	2	1	0	23/24	95.8
Zhang et al. [9]	2	2	2	2	1	2	2	2	2	2	2	2	2	25/26	96.0
He et al. [11]	2	2	2	2	0	1	2	2	2	2	2	1	1	21/24	87.5
Chen et al. [19]	2	2	2	2	0	0	2	2	2	2	2	1	1	20/22	90.1

∗Note: significance evaluation: 2—yes; 1—limited detail; 0—no; NA: not applicable.

**Table 2:** Participants' or models' characteristic.

Authors	Condition/category	Number of participants/models	Gender		Anthropometric data
			Male	Female	
Dumas et al. [10]	Postsurgical patients	2	NM	NM	Age: 30 and 35
Abolaeha et al. [12]	Postsurgical patients	NM	NM	NM	NM
Salmingo et al. [1]	Postsurgical patients	3	3	0	Age: 16, 15 and 14
Wang et al. [13]	Postsurgical patients	10	10	0	Age: adolescent Height: 162 cm-172 cm Weight: 47 kg-64 kg
Driscoll et al. [6]	Spine finite element model	1	NM	NM	NM
Salmingo et al. [2]	Pre- and postsurgical patients	6	NM	NM	Age: adolescent
Little et al. [3]	Postsurgical patients	8	NM	NM	Age: adolescent
Abe et al. [14]	Postsurgical patients	20	1	19	Age: adolescent
Wang et al. [15]	Presurgical patient	1	1	0	Age: NM Height: 168 cm Weight: 65 kg
Clin et al. [16]	Postsurgical patients	5	0	5	Age: adolescent
Balamurugan et al. [17]	Spine finite element model	1	NM	NM	NM
Guan et al. [18]	Postsurgical patients	1	NM	NM	Age: 11
Zhang et al. [9]	Presurgical patients	1	0	1	Age: 14 Weight: 45 kg
He et al. [11]	Normal spine	1	1	0	Age: 40 Height: 170 cm Weight: 60 kg
Chen et al. [19]	Postsurgical patients	1	0	1	Age:15

Note: NM-not mentioned.

**Table 3:** Variables of FEA studies on the corrective mechanism of spine deformity.

Authors	Software(s)	Element type	Geometrical model	Loading and boundary conditions	Type of material	Mechanical properties
Dumas et al. [10]	Ansys 6.0.	(i) Vertebra: beam element (ii) pelvic: beam element (iii) ligament: tension-only cable elements (iv) articular facets: surface contact element	A patient-specific FE model of interverbal disc constructed from CT image.	Displacement: between the bending test measurements and the standing position measurements, 3D motion of T1 in relation to the pelvis was estimated.	Screws and rod: elastoplastic materials	(i) Augmented bending stiffness (about *K*_*f*_ × 60) from T5 to T9; (ii) augmented torsion stiffness (about *K*_*t*_ × 80) from T6 to L5
Abolaeha et al. [12]	Abaqus 6.11-1	(v) Vertebral and intervertebral disc: linear hexahedral (vi) Hooks and screw: quadratic tetrahedral element	A previous patient-specific FE model of vertebral and interverbal disc constructed from X-ray image and CT scan	During the loading and spine growth simulation processes, the inferior extremity of L5 was constrained in all degrees of freedom. Each vertebra is subjected to a dispersed load.	Rod: stainless steel	*E* = 190 GPa*ν* = 0.4
Salmingo et al. [1]	Computed tomography (CT), Solidworks 2010, ANSYS 11.0	10 node tetrahedral solid elements	A patient-specific FE model of spine constructed from CT image.	Forces, *Fi* set with initial values. The coordinates of the screws were rearranged so that the most superior screw is parallel to the *z*-axis.	Rod: titanium alloy (JIS T 7401-3)	E = 105 GPa yield stress (*σY*) = 900 MPa yield strain (*εY*) = 8.57 × 10^−3^ hardening coefficient (*H*) = 2.41 GPa
Wang et al. [13]	Radiographic software, ADAMS 2005 software (Mechanical Dynamics)	NM	Previously developed FE model of thoracic spine.	NM	Pedicle screw: titanium rod: titanium	*E* is 15 to 20 times higher than that of spinal cortical bone.
Driscoll et al. [6]	ANSYS 130.0 APDL	NM	A patient-specific FE model of vertebral and interverbal disc constructed from CT image.	To regulate and measure movement, all bodies assigned multiple coordinate systems centred on their geometric centre of mass.	Screw: titanium (Ti 6Al-4 V, grade 5) rod: cobalt chrome	Pedicle screw: *E* = 11 GPa Rod: *E* = 213 GPa
Salmingo et al. [2]	Solidworks 2010, ANSYS 11.0	10 node tetrahedral solid elements	Three-dimensional FE model of rod geometries before surgery.	Before surgery. Zero force *Fi* (*i* = no. of screws) was applied to the corresponding location of each screw on the rod geometry.	Polyaxially pedicle screws and implant rods: titanium	*E* = 105 GPa Yield stress (*σY*) = 900 MPa Yield strain (*εY*) = 8.57 × 10 − 3 Hardening coefficient (*H*) = 2.41 GPa
Little et al. [3]	Computed tomography (CT), ABAQUS 6.9-1, Python 2.5	(i) Screw: 8 node brick (ii) Rod: 8 node brick and 2 node rigid beam	A patient-specific FE model with ribcage and Osseo ligamentous spine	A “no separation” normal contact and frictionless tangential contact definition were defined between the both surface of the rod and the screw head.	Screw: titanium alloy Rod: titanium alloy	Screw: *E* = 108 GPa Rod: *E* = 108 GPa Coulomb friction, *ν* = 0.3 Yield stress = 390 MPa
Abe et al. [14]	Solidworks 2010, Aquilion 64 CT scanner, ANSYS 11.0	10 node tetrahedral solid elements	A patient-specific model of rod geometry constructed from CT image.	NM	Rod: titanium rod (Ti6Al7Nb)	*E* = 105 GPa Yield stress (sY) = 900 MPa Yield strain (*εY*) = 8.57 × 10 − 3 Hardening coefficient (*H*) = 2.41 GPa
Wang et al. [15]	Computed tomography (CT), ANSYS ICEM-CFD	Hexahedron element	A patient-specific FE model of the spine constructed from CT image. -Thoracic spine, the lumbar spine and sacrum.	The upper lamina terminals of T1 were subjected to a fixed loading force of 300 N, which simulated upper body gravity.	Pedicle screw and rod elastoplastic materials	Ligaments elasticity coefficient
						Anterior longitudinal, *E* = 21.34 N/mm Posterior longitudinal, *E* = 36.42 N/mm, interspinous, *E* = 19.96 N/mm, ligamentum flava, *E* = 26.78 N/mm Supraspinal. *E* = 0.04 N/mm
Clin et al. [16]	ANSYS 14.5	NM	A patient-specific FE model of the spine to pelvis	NM	Screw: titanium alloy Rod: cobalt chrome	*E* = 213 GPa *E* = 113 GPa
Balamurugan et al. [17]	MIMICS 14.0 software, ANSYS 18.0	NM	A patient-specific FE model of thoracolumbar constructed from CT image	All degrees of freedom were limited in the L5 vertebra. Assuming the patient's weight is 800 N (80 kg), apply a compressive force of 50 N all along *z*-axis to T1. Vertebra.	Rod: titanium	Cortical bone: *E* = 1200 MPa *ν* = 0.26 Bone posterior: *E* = 3500 MPa *ν* = 0.25
Guan et al. [18]	Materialise mimics 19.0, Leuven, Abaqus,	Hexahedral elastic elements	A patient-specific FE model of the thoracic spine lumbar vertebrae constructed from CT image	T1 was limited to transverse plan movements.	Elastoplastic spine model	Posterior structure: *E* = 3500 MPa *ν* = 0.25 = 1000 kg/m^3^
Zhang et al. [9]	Solidworks 2020, Ansys Workbench 19.0	Tetrahedral elements	A patient-specific FE model of the lumbar spine constructed from CT image	Apply a moment of 10 nm in the planes on the upper surface of the L1 vertebral body to simulate flexion, extension, left and right bending, left and right rotation.	Elastoplastic spine model	Cortical bone: *E* = 12 GPa *ν* = 0.3 Cancellous bone: *E* = 100 MPa *ν* = 0.3 Annulus fibrosis: *E* = 4.2 MPa *ν* = 0.453 Nucleus pulposus: *E* = 1 MPa *ν* = 0.499
He et al. [11]	Mimics 19.0, ANSYS 15.0	Solid 187 tetrahedral elements	Three-dimensional finite element (FE) model of intervertebral disc and pedicle screw & rod system (PSRS).	500 N applied to the models for directions of flexion, extension, lateral bending, and axial rotation	Screw and rod: titanium alloy	Cortical bone: *E* = 12 GPa Poisson′s ratio = 0.3 Cancellous bone: *E* = 100 MPa Poisson′s ratio = 0.2 Annulus fibrosis: *E* = 4.2 MPa Poisson′s ratio = 0.450 Titanium alloy: *E* = 110 GPa Poisson′s ratio = 0.25
Chen et al. [19]	CT scan, Solidworks	NM	Three-dimensional finite element (FE) model of the spine from CT, pedicle screw, and rod system.	NM	Rod: titanium alloy	Cortical bone *E* = 14 Pa Poisson′s ratio = 0.3 Cancellous bone *E* = 500 MPa Poisson′s ratio = 0.3

∗Note: *E*: Young modulus; *ν*: Poisson ratio; *K*: the strength coefficient; NM: Not mentioned.

**Table 4:** Data extraction on the effect of Cobb angles from the reviewed articles.

Authors	Category	Plane	Situation/ Zone	Cobb Angle		Outcome Measures	Parameter Output			Findings
Dumas et al. [10]	Simulation of clinical data and post-operative measurements comparison & rod rotation analysis	Lateral, Sagittal, Axial	Scheuermann hyper kyphosis Idiopathic scoliosis	50° 58°		Rod rotation (°)	Lateral rotation= - Sagittal rotation= Mean :4° = Max: 9° Axial rotation= - Lateral rotation= Mean :3° = Max: 7° Sagittal rotation = Mean :4° = Max: 9° Axial rotation = Mean :5° = Max: 11°			The surgeon's experience was consistent with models of two clinical situations of hypokyphosis and scoliosis. Follow-up: NM.
Abolaeha et al. [12]	Spinal growing rod analysis	Sagittal & Axial	Cycle of Adjustment period Initial 1^st^ growth 2^nd^ growth 3^rd^ growth 4^th^ growth	Before 37° 42° 40° 39° 49°	After 28° 34° 33° 37° 40°	Magnitude of force	Compressive force (N) 362N 669N 942N 1215N 1454N	Rod Displacement(mm) 5 10 17 20 30		The rod length was changed until the desired Cobb angle was achieved, which was decreased from an initial value of 37° to 28°. This necessitated a 5 mm lengthening of the rod, resulting in a correction force of 362 N. Follow-up: 2 years
Salmingo et al. [1]	The three-dimensional corrective forces analysis	Frontal (x-z plane)	Patient 1 Patient 2 Patient 3	Before 57° 59° 68°	After 13° 28° 18°	3D Forces(N), Stress, Strain Distribution	Only the rod geometry before and after the surgical treatment was used to analyse the distributions of forces that distorted the implant rod.			The highest force acting on each patient's screw ranged from 198 to 439 N. The force magnitude was clinically acceptable. The maximal forces were generated at each patient's lowest fixation level of vertebra. Follow-up: NM
Wang et al. [13]	The corrective forces & bone-screw forces analysis	Sagittal & Axial	NA	Sagittal curve: 5.3° Vertebral axial: 4°- 8°		Resultant Screw force(N)	TCF magnitudes vs resultant screw force magnitudes associated with monoaxial, dorsoaxial and polyaxial pedicle screw.			True corrective forces were 50±30N on average. For monoaxial, dorsoaxial and polyaxial screws, the average bone-screw forces were 229±140N, 141±99N, and 103±42N, respectively; the average EF magnitudes were 205±136N, 125±93N, & 65±39N respectively. Follow-up: NM.
Driscoll et al. [6]	The three-dimensional corrective force analysis	Transverse, Axial, & Sagittal	NA	Right thoracic: 73° Proximal thoracic: 42°		Screw pull-out force	T3 T4 T5 T6 T7 T8 T9 T10 T11 T12 L1	0 1000N ≈350N 300N - 349N 0 0 300N - 349N <200N ≈350N >800N 0		Over the course of the surgical process simulation, stress in intervertebral discs discovered between instrumented vertebrae averaged 3.95MPa. Follow-up: NM
Salmingo et al. [2]	The three-dimensional corrective forces analysis	Sagittal	Patient 1 Patient 2 Patient 3 Patient 4 Patient 5 Patient 6	Before 76° 75° 57° 68° 83° 59°	After 27° 26° 13° 18° 14° 28°	Pull-out and push-in force	The screw density and implant implantation arrangement all contributed to a higher degree of correction. This shows that if more implants are put closer together, vertebrae can be easily altered.			Forces of correction are unrelated. Although increasing the number of implant screws reduced the magnitude of corrective forces, it did not result in a higher degree of correction. Follow-up: NM
Little et al.[3]	The three-dimensional corrective forces analysis	Coronal	Patient 1 Patient 2 Patient 3 Patient 4 Patient 5 Patient 6 Patient 7 Patient 8	Before 52° 51° 44° 53° 40° 42° 42° 53°	After 23° 18° 14° 25° 10° 7° 13° 34°	Degree of deformity correction, Compressive force profile	-3 -2 -1 0 1 2 3	400N 580N 675N 660N 550N 470N 320N		Endplate-to-endplate contact was seen on adjacent endplates of one or more intervertebral disc spaces in the instrumented curve after the surgical loading procedures, according to patient model predictions. Follow-up: NM
Abe et al. [14]	The corrective force estimation	NM	NA	Thoracic: 53°- 74°		Push out or push in forces	Convex	F1 F2 F3 F4 F5 F6 F7	113N 31N 48N 55N 52N 34N 123N	The concave side corrective force is four times greater than in convex side. Follow-up: NM
							Concave	F1 F2 F3 F4 F5 F6 F7	424N 105N 169N 218N 214N 142N 466N	
							Flexion	L2-L3 L3-L4 L4-L5	3.28°-.4° 3.06°-1° 3.58°-1°	Axial compression- The rod was the part that was subjected to the most stress Flexion- the stress was centred on proximal pedicle screws. Extension and lateral bending- an osteotomized L1 vertebra bore the greatest stress on the model. Follow-up: NM
							Extension	L2-L3 L3-L4 L4-L5	2.3°-3.3° 1.18°-2.3° 2.56°-4°	
Wang et al. [15]	The stress-strain analysis	Coronal	NA	Thoracolumbar: 53°		The ranges of motion (ROM)	Lateral Bending	L2-L3 L3-L4 L4-L5	3.31°-5.0° 3.33°-4.3° 2.08°-4.01°	
Clin et al. [16]	Pedicle screw design & Load-Sharing Capacity analysis	Transverse & coronal	NA	Thoracic: 53°-85°		Derotation force, axial torque	The average post-instrumentation force sustained by high and low-density implant patterns with varied pedicle screw design configurations was recorded, as well as the peak force experienced during surgery simulation.			Increased degrees of freedom in the screw head limit the screw's ability to cure coronal deformity while lowering bone-screw forces. Follow-up: 10 years
Balamurugan et al. [17]	Effect on spine deformity correction	NM	NA	NM		Stress distribution	T5 T6 T7 T8 L1 L2 L3 L4 L5	<0.5MPa <0.5MPa <0.5MPa 300 – 349MPa 0-0.5MPa 0.5-1MPa >1.5MPa >1.5MPs >1.5MPa		After surgery, the stress concentration is highest near the end of the lumber area. Follow-up: NM
Guan et al. [18]	The three-dimensional corrective forces analysis	Coronal, sagittal and horizontal	(i) Forward bend (ii) Stretch (iii) Side bender (iv) Twists	Thoracic: 14°-36° Lumbar: 10°-17°		Stress	As the 3D corrective forces increased, the cobb angle of the thoracolumbar section reduced, as did the rotation angle of the vertebra. The combined force correction effects were higher.			The objective functions were each lowered by 58%, 52%, and 63 percent. On the convex side of the highest displacement of the vertebral body, the optimal corrective forces point was found. Follow-up: NM
Zhang et al.[9]	Stress distribution	Coronal, sagittal and frontal	NA	Frontal: 43° Lumbar: 45°		Stress distribution	Stress is concentrated on the lumbar vertebral body during flexion loading, with an unequal stress distribution on the left anterior side of the vertebral body (concave side). Stress in the lumbar spine is localised primarily at the pedicle of the vertebral arch and the lamina of the vertebral arch during extension load.			Under all loads, the range of motion (ROM) is reduced. Flexion loads cause a greater distribution of vertebral concave stress. The stress is concentrated in the L3 vertebral arch. Follow-up: NM
He at al. [11]	The three-dimensional corrective forces analysis	Coronal, sagittal and horizontal	NA	NM		Stress shielding rate	FEA analysis of the new improved spinal correction system ISCS to determine its stability and biomechanical features, as well as a comparison of the ISCS to the pedicle screw and rod system (PSRS).			Maximum stress L2 vertebral body & L1/2 and L2/3 discs in PSRS were smaller than in ISCS. PSRS and ISCS have identical maximum stress in lateral bending and axial rotation directions. Follow-up: NM
Chen at al [19]	The pedicle screw placement strategies	Sagittal	(a) All segments have pedicle screws placed. (b) Pedicle screws were implanted in all of the concave side's segments, with interval screws inserted in the convex side. (c) Both side alternate screws (d) instruments on both sides of the interval screws (e) interval and alternate screws instrumentation in each side	Thoracic: 43°		Interaction force	113N 113N 289N 172N 172N			Densities of pedicle screws and screw-placement techniques have little influences in the curve correction. Strategy E has better biomechanics properties for surgery. Follow-up: NM

## Data Availability

The data used to support the findings of this study are available from the corresponding author upon request.
